# Not All Critically Ill Obese Patients Are the Same: The Influence of Prior Comorbidities

**DOI:** 10.5402/2012/743978

**Published:** 2012-11-04

**Authors:** Adam Rahman, Renee D. Stapleton, Daren K. Heyland

**Affiliations:** ^1^Division of Gastroenterology, Department of Medicine, McMaster University, Hamilton, ON, Canada N6A 4V2; ^2^Division of Critical Care Medicine, Department of Medicine, Niagara Health System, Hamilton, ON, Canada; ^3^Division of Pulmonary and Critical Care Medicine, Department of Medicine, University of Vermont, Burlington, VT 05405, USA; ^4^Clinical Evaluation Research Unit, Kingston General Hospital, Kingston, ON, Canada K7L 2V7; ^5^Department of Community Health and Epidemiology, Queen's University, Kingston, ON, Canada K7L 2V7; ^6^Department of Medicine, Queen's University, Kingston General Hospital, Kingston, ON, Canada K7L 2V7

## Abstract

*Purpose. *Data suggest that obesity in critical illness is associated with improved outcomes. We postulate that these findings may be influenced by preillness comorbidities. We sought to determine if critically ill obese patients without significant comorbidity had improved mortality compared to obese patients with multiple comorbidities. *Materials and Methods*. We analyzed data from a prospective observational study conducted in 3 tertiary ICUs. Severely obese (body mass index ≥30) adults in the ICU for ≥24 hours were identified and classified into limited comorbid illnesses (0-1) or multiple comorbidities (≥2). The primary outcome was the odds ratio (OR) of mortality at day 28. Important secondary outcomes were ICU length of stay and ICU free days in the first 28 days. *Results*. 598 patients were enrolled; 183 had BMI ≥30. Of these, 38 had limited comorbidities and 145 had multiple comorbidities. In unadjusted analyses, obese patients with multiple comorbidities were 4.70 times (95% CI 1.07–20.6) as likely to die by day 28 compared to patients with limited comorbidities (*P* = 0.04). After stratifying by admission diagnosis and adjusting for APACHE II score, the influence of comorbidities remained large and trended toward significance (OR 4.28, 95% CI 0.92–20.02, *P* = 0.06). In adjusted analyses, obese patients with multiple comorbidities tended to have longer ICU duration (3.06 days, SE 2.28, *P* = 0.18) and had significantly fewer ICU free days in the first 28 days (−3.92 days, SE 1.83, *P* = 0.03). *Conclusions*. Not all critically ill obese patients are the same. Those with less comorbidity may have better outcomes than those with multiple comorbidities. This may be important when considering prognosis and discussing care with patients and families.

## 1. Introduction

Obesity is excessive body fat. Various anthropometric classifications exist to define obesity and classify severity, based on weight, height, and waist circumference [1]. Recent studies suggests that obese patients (body mass index [BMI > 30]) with critical illness have equivalent or lower mortality rates than equally sick, nonobese patients [2–10]. These observations are supported by a meta-analysis which suggested that patients with a BMI >40 had decreased hospital mortality compared to normal weight patients, although this did not reach statistical significance (relative risk [RR] 0.83, 95% confidence interval [CI] 0.66–1.04) [9]. Because we intuitively might expect a mortality increase in the obese population, this phenomenon has been coined the “obesity paradox” [8].

Reasons for the lack of mortality increase in extremely obese patients are unknown. However, a recent study found that obese patients with acute lung injury have lower levels of several proinflammatory cytokines (interleukin-6, interleukin-8, and surfactant protein D) [11], raising the possibility that obese may develop a reduced inflammatory response in critical illness. Another hypothesis is that increased energy stores and increased lean body mass in obese patients may provide protective effects.

Classic anthropometric systems, such as body mass index (BMI), do not necessarily predict quality of life or obesity-related health complication [1, 12]. However, when obesity is associated with comorbid disease and functional limitation, patients are at increased risk for mortality and a broad spectrum of other health risks [1, 13]. Because the morbidity of obesity is often dependent on the presence of associated disease, we postulate the subpopulation of critically ill obese patients *without* significant comorbid disease are most likely to have the best outcome. Moreover, the previous studies examining the relationship between mortality and obesity in critically ill patients often only rely on severity of illness markers that include a few comorbid illness, such as Acute Physiology And Chronic Health Evaluation (APACHE) II [14] and Simplified Acute Physiology Score (SAPS) II scoring systems [15] (see Table 1). Only two studies corrected for comorbidities in a comprehensive manner. Sakr et al. [4] performed COX regression analysis for comorbid disease including chronic obstructive pulmonary disease, congestive heart failure, cancer, and diabetes mellitus only. When adjusting for comorbid illnesses they showed no significant mortality differences between obese and normal weight obese patients. Memtsoudis et al. [8] 2011 also performed regression analysis for comorbid illness, using the Deyo-comorbidity index. When adjusting for comorbidity burden, they showed significant mortality reduction in surgical obese critically ill patients with acute lung injury, compared to nonobese patients.

Our primary hypothesis is that not all obese critically ill patients will have the same outcome and those with a more significant burden of pre-ICU comorbid illness will have a worse outcome than those with no or less significant comorbid illness. We analyzed an existing database with anthropometric measures, clinical outcomes, and biomarkers collected in a prospective study [16] to determine if signals are present to suggest if obesity with limited comorbidity is associated with better outcomes compared to those with multiple comorbidities. The answer to this question has significant impact on prognosticating and may assist in planning care for such patients. 

## 2. Methods

We conducted a prospective multicenter observational study in three tertiary care ICUs for the primary purpose of evaluating a novel diagnostic marker for sepsis [16]. In the original study, all patients admitted to the ICU and expected to stay more than 24 hours were included. We excluded those admitted for routine cardiac monitoring (i.e., elective surgery), overdoses, and pediatric patients (<18 years of age). Herein, we report a secondary analysis examining the relationship between obesity and subsequent outcomes. Obese patients (obese class I, II, and III) defined as a body mass index (BMI) of ≥30 were identified [13]. Local institutional research ethics boards approved the protocol and informed consent was obtained prior to enrolment. The clinical management of patients was determined by the clinical team caring for the patient as per the clinical protocols operational in each respective ICU. 

### 2.1. Data Collection

Baseline demographics, past medical history, and reasons for ICU admission were obtained from patients or their charts. Necessary variables were recorded to calculate APACHE II score [14] on admission and SOFA scores [17] daily until day 28, death or discharge from the ICU. Comorbidities were abstracted from the hospital record; a simple taxonomy (shown in the Appendix) was used to record the presence or absence of comorbidities. The maximum number of comorbidities entered into the database was 5. Blood samples were collected for analysis in the morning following enrolment and each subsequent ICU day until discharge, death, or a maximum of 10 days. Plasma was analyzed for inflammatory and coagulation markers using the following assays: protein C (PC) [MDA Protein C assay kit, Organon Teknika Corporation, Durham, NC, USA]; antithrombin (AT) [MDA Antithombin III assay kit, BioMerieux, Inc. Durham, NC, USA]; D-Dimer [MDA D-Dimer assay kit, Organon Teknika Corporation, Durham, NC, USA]; IL-6 [Bender Medsystems ELISA kit-Cat BMS-213 (Bender Med systems Inc., Burlingame, CA, USA)], PCT [BRAHMS PCT LIA assay, (Hennigsdorf, Germany)]. C-reactive protein (CRP), fibrinogen, and cholesterol levels were all analyzed at local institutions according to standard laboratory operating procedures. 

### 2.2. Outcome Measurements

The primary outcome for this study was 28 day ICU mortality. Important secondary outcomes were ICU free days in the first 28 days and number of days in the ICU. Additional outcomes included differences in inflammatory markers between the two groups, as well as maximum and delta SOFA scores. Delta SOFA score was calculated by subtracting the maximal SOFA score from the baseline score [17].

### 2.3. Data Analysis

We examined the frequency of comorbidities in our subpopulation (see Figure 1). Since there were too few patients with no comorbidities, we combined patients with “0” and “1” comorbidities together to form a group with “limited” comorbidities and compared them to patients with 2 or more comorbidities (multiple group). Patient characteristics, clinical outcomes, and biomarkers were compared between obese patients with limited and multiple comorbidities. Categorical variables were described as counts and percentages and compared by Chi-square tests whereas continuous variables were described as means with standard deviations or medians with intraquartile ranges and compared by the Wilcoxon-Mann-Whitney test. Logistic regression was used to calculate the unadjusted odds ratio (OR) and 95% confidence intervals (CI) of 28 day mortality and linear regression was used to calculate unadjusted estimate of days on mechanical ventilation, days in the ICU and ICU free days. To account for differences in covariates that were significantly different between groups, we also examined these clinical outcomes for obese patients with multiple comorbidities versus limited comorbidities after stratifying for primary admission diagnosis and adjusting for APACHE II score (which includes age in its calculation). 

## 3. Results

### 3.1. Baseline Characteristics

598 patients were enrolled in the original study. We identified 183 patients with BMI ≥ 30; 38 had limited comorbidities (0-1) and 145 had multiple comorbidities (≥2). Baseline characteristics of the two groups are shown in Table 2. Average age was 56.8 years in the obese group with limited comorbidities, compared to 66.1 years for the multiple comorbidities group (*P* < 0.001). There were significant differences in the primary admission diagnoses with more patients admitted with respiratory conditions and fewer with trauma in the multiple comorbidities group (*P* = 0.02). The average APACHE II score was 17.5 for obese patients with limited comorbidities (0-1) and 22.0 for the multiple comorbidity group (*P* = 0.04). There were no differences in time in hospital prior to admission to the ICU, or other markers from day 1 of admission, including heart rate, temperature, *P*_*a*_O_2_/*F*_*i*_O_2_  (*P*/*F*) ratio, and white cell count (WBC).

### 3.2. Outcomes

In Table 3, we show the unadjusted outcomes of the 2 groups. Of the 38 obese patients with limited comorbidities, 2 (5.3%) (2/38) died by day 28, versus 20.7% (30/145) patients in the multiple comorbidities group (*P* = 0.03). ICU free days in the first 28 days were greater in the limited comorbidities group compared to the multiple comorbidities group; 24.5 versus 20.0 days, respectively (*P* = 0.01). The number of days in ICU was lower in the limited comorbidities group compared to the multiple comorbidities group (3.0 versus 6.0, *P* = 0.04). There were differences in maximum SOFA score, 7.5 for obese patients in the limited comorbidities group, and 9.0 for obese patients with multiple comorbidities (*P* = 0.04). Delta SOFA scores between limited and multiple comorbidity groups were 1.5 versus 2.0, respectively (*P* = 0.07).

In an unadjusted analysis, obese patients with multiple comorbidities were 4.70 times (95% CI 1.07, 20.6) as likely to die by day 28 compared to patients with limited comorbidities (*P* = 0.04). After stratifying by primary admission diagnosis and adjusting for APACHE II score, the influence of comorbidities was still large but just short of conventional statistical significance (OR of death by day 28 = 4.28, 95% CI 0.92, 20.02, and *P* = 0.06).

Obese patients with multiple comorbidities tended to have a longer ICU duration compared to patients with limited comorbidities (2.92 days, standard error [SE] 2.02, and *P* = 0.15). After stratifying for primary admission diagnosis, and adjusting for APCAHE II scores, there was still a trend towards increased duration of stay in ICU in the multiple comorbidities group (3.06 days, SE 2.28, and *P* = 0.18). No differences were noted between the two groups for days on mechanical ventilation in either the adjusted or unadjusted analysis (data not shown).

Obese patients with multiple comorbidities had 4.5 (SE 1.78) fewer ICU free days in the first 28 days compared to patients with limited comorbidities (*P* = 0.01). After stratifying for primary admission diagnosis and adjusting for APACHE scores, there was still a significant reduction in ICU free days in the multiple comorbidities group (−3.92 days, SE 1.83, and *P* = 0.03).

We also compared various markers of systemic inflammation, coagulation, and metabolism between the two groups (see Table 4). No significant increases were observed in levels of D-dimer, protein C, antithrombin, procalcitonin, CRP, fibrinogen, IL-6, triglycerides, or in HDL/LDL cholesterol.

## 4. Discussion

Our study specifically examines the relationship between comorbidities and clinical outcomes in critically ill obese patients. As compared to critically ill obese patients with limited comorbidities (0 to 1), our results suggest patients with multiple comorbidities (2 or more) are about 3-4 times more likely to die and have fewer ICU free days in the first 28 days. No differences were noted in days in ICU or days on mechanical ventilation. There were no differences between the groups in levels of biomarkers. 

Previous data suggest that the survival of obese critically ill patients is at least as good as, and may be better than, normal weight patients [2–9], a finding which has been coined the “obesity paradox” [8]. Recently, Martino et al. [10] analyzed data from a multicenter international observational study of ICU nutrition practices that occurred in 355 ICUs in 33 countries during 2007–2009. They compared extremely obese (BMI ≥ 40) ventilated patients to normal weight patients in terms of duration of mechanical ventilation (DMV), ICU LOS, hospital LOS, and 60-day mortality. They concluded that extreme obesity is not associated with increased mortality, although severe obesity (BMI ≥ 60) was associated with longer time on mechanical ventilation and in the ICU. These authors [10] comment that extremely obese patients may have a lower threshold for ICU admission compared to normal weight patients, meaning the disease severity is less than perceived, thus accounting for an apparent benefit. In another recent study, a nationwide inpatient sample database was analyzed in the United States for each year between 1998 and 2007 (over 9 million patients). Patients were included if they underwent a surgical procedure and had a diagnosis of respiratory insufficiency or acute respiratory distress syndrome following surgery. In-hospital mortality for obese patients (BMI > 30) was significantly lower compared to nonobese patients (5.45% versus 18.72%), maintaining statistical significance with multi-variable analysis [8].

Reasons for this reported mortality benefit in critically ill obese patients are not known. One explanation might be an alteration in the inflammatory response as suggested by a recent study that reported that obese patients with acute lung injury have lower levels of several proinflammatory cytokines including surfactant proteins, IL-6 and IL-8 [11]. In our study, however, serum inflammatory markers and activated coagulation measures between obese patients with limited and multiple comorbidities were not different. Thus, we cannot explain apparent differences in clinical outcomes by these different biochemical pathways, although our sample size, in regards to this analysis, was limited. 

Our results suggest that obese patients with limited comorbidities may have decreased mortality and more ICU free days compared to those with multiple comorbidities. While some of our results did not reach statistical significance, we were limited by small sample size and considerable heterogeneity between the two groups. These signals that obesity with limited comorbidity may be associated with better outcomes add another level of complexity to the paradox of critical illness and obesity. 

As BMI was similar between the limited and multiple comorbidity groups, our results seem not to be associated with the degree of obesity. This finding supports the notion that traditional anthropometric classification of obesity, while useful in population models, may not provide the necessary clinical information and functional limitation that apply to individual obese patients [18]. In fact, the morbidity of obesity is so dependent on the presence of associated diseases, that many cardiovascular risk scoring systems do not take into account anthropometric measures of obesity [12]. Our findings of differences in clinical outcome that are based on the burden of comorbidity and not on the severity of obesity suggest that adoption of additional clinical measures of obesity, beyond traditional classification, may be necessary in critically ill patients. Sharma and Kushner [1] recently proposed a five-level classification system that progressively grades obesity on clinical and functional measures. He and his colleagues demonstrated that as functional status declines, subsequent mortality rates increase thus validating this concept of functional obesity [18]. Integration of these types of classification schemas into practice may allow us to better treat and prognosticate critically ill patients who are obese and direct future research.

The limitations of our work include our definition of comorbidity. While the absence or relative absence of comorbidity intuitively defines a lower comorbidity group, the 0-1 definition in our classification system has not been independently validated in obese patients. There are well validated methods of quantifying comorbidity, such as the Charlson comorbidity Index (CCI) [19]. Because the database system was limited to simple taxonomic counting of a maximum of 5 comorbidities, however, calculation of CCI or other validated methods of quantifying comorbidity was not possible. Moreover, it is possible that one group had more of a specific comorbidity that predisposed to a better or worse outcome. A further limitation of our work is our limited sample size which resulted in imprecise estimates of effect. However, despite this limited sample, the observed differences were large and clinically important.

## 5. Conclusion and Future Direction

There is a growing body of literature suggesting obesity may have protective effects in critical illness. However, critically ill obese patients are a heterogeneous group and our data suggest another level of complexity to the obesity paradigm. We observe that obese patients with lower comorbidity may have improved outcomes, including trends for improved mortality at 28 days and increased ICU free days in the first 28 days as compared to obese patients with multiple comorbidities. 

The prevalence of obesity in the critical care population is increasing, mirroring changes in the general population. These findings are important when considering prognosis and discussing care with patients and families. Given the challenges in providing care to this population, much more work needs to be done in this area. We would advocate for a large, prospective study to further delineate the association of obesity with patients with critical illness, with particular focus on nutritional status and characterizing obesity with clinical/functional staging and validated measures of comorbidity. 

## Figures and Tables

**Figure 1:** Distribution of comorbidities.

**Table 1:** Studies examining mortality in obese critically ill patients and the adjustments for co-morbid illness.

Author	BMI of obese patients and no.	Study design	Findings	Adjustments for co-morbidity in multivariate analysis
Ray et al. (2005) [3]	BMI ≥ 30, *n* = 237	Retrospective. (ALI patients)	No mortality difference.	APACHE II only
Frat et al. (2008) [6]	BM ≥ 35, *n* = 121	Matching.	No mortality difference with obesity but difficulty with intubation and stridor.	SAPS II only
Sakr et al. (2008) [4]	BMI ≥ 30, *n* = 505	Retrospective.	No difference in mortality in but increased LOS.	SAPS II Cancer, CHF, COPD, and DM
Aldawood et al. (2006) [2]	BMI ≥ 30, *n* = 971	Retrospective.	Lower mortality.	APACHE II Chronic respiratory illness.
O'Brien et al. (2006) [5]	BMI ≥ 30, *n* = 458	Retrospective. (ALI patients)	Lower mortality.	SAPS II only
Garrouste-Orgeas et al. (2004) [7]	BMI ≥ 30, *n* = 232	Retrospective. (surgical patients)	No mortality difference.	APACHE II only
Memtsoudis et al. (2012) [8]	BMI ≥ 30	Retrospective. (surgical/ARDS)	Lower mortality in obese patients.	Deyo co-morbidity index
Martino et al. (2011) [10]	BMI ≥ 40, *n* = 524	Retrospective. (nutrition survey)	No mortality difference with obesity but longer time on mechanical ventilation and in ICU.	APACHE II only

**Table 2:** Patient characteristics.

	0-1 co-morbidity	2 or more co-morbidities	*P* values
	(*n* = 38)	(*n* = 145)	
Age (years)	56.8 [46.4 to 64.4]	66.1 [55.1 to 72.9]	**<0.001**
Sex			
Male	21 (55.3%)	71 (49.0%)	0.49
Admission			0.45
Medical	21 (55.3%)	90 (62.1%)	
Surgical	17 (44.7%)	55 (37.9%)	
Primary admission diagnosis			**0.02**
Cardiovascular/vascular	4 (10.5%)	13 (9.0%)	
Respiratory	5 (13.2%)	44 (30.3%)	
Gastrointestinal	9 (23.7%)	27 (18.6%)	
Neurologic	4 (10.5%)	9 (6.2%)	
Sepsis	2 (5.3%)	5 (3.4%)	
Trauma	7 (18.4%)	6 (4.1%)	
Metabolic	1 (2.6%)	4 (2.8%)	
Postoperative conditions	2 (5.3%)	23 (15.9%)	
Renal	1 (2.6%)	11 (7.6%)	
Orthopedic	3 (7.9%)	3 (2.1%)	
Family history diabetes			0.96
Yes	6 (15.8%)	19 (13.1%)	
No	12 (31.6%)	37 (25.5%)	
Unknown	20 (52.6%)	89 (61.4%)	
APACHE II score	17.5 [13.0 to 24.0]	22.0 [15.0 to 26.0]	**0.04**
Baseline SOFA	5.0 [4.0 to 8.0]	7.0 [5.0 to 9.0]	0.08
No. of days in hospital prior to ICU admission	0.4 [0.1 to 0.9]	0.3 [0.0 to 2.6]	0.85
Waist circumference (cm)	112.5 [106.0 to 124.0]	117.0 [109.0 to 125.0]	0.42
Hip circumference (cm)	116.0 [106.0 to 125.0]	114.0 [107.0 to 126.0]	0.82
Height (cm)	171.0 [ 160.0 to 178.0]	166.0 [160.0 to 174.0]	0.12
Weight (Kg)	102.2 [93.0 to 112.2]	96.0 [85.0 to 108.0]	0.07
BMI	35.5 [31.9 to 39.1]	33.8 [31.5 to 38.7]	0.29
*Data on ICU admission Day *			
Heart rate (per minute)	111.0 [94.0 to 122.0]	100.0 [86.0 to 118.0]	0.09
Temperature (degrees Celsius)	37.9 [37.3 to 38.4]	37.8 [37.0 to 38.5]	0.54
Respiratory rate (per minute)	22.5 [18.0 to 27.0]	22.0 [18.0 to 29.0]	0.98
PF ratio	210.6 [122.0 to 278.6]	170.6 [101.4 to 240.0]	0.15
WBC	12.6 [9.9 to 16.4]	11.7 [8.2 to 17.4]	0.49

**Table 3:** Clinical outcomes.

	0-1 co-morbidity (*n* = 38)	2 or more co-morbidities (*n* = 145)	*P* values
Discharged alive from ICU by day 28	36 (94.7%)	112 (77.2%)	**0.02**
Maximum SOFA score	7.5 [5.0 to 11.0]	9.0 [6.0 to 13.0]	**0.04**
Delta SOFA score	1.5 [0.0 to 3.0]	2.0 [1.0 to 5.0]	0.07
Number of days on MV	2.0 [1.0 to 5.0]	4.0 [2.0 to 7.0]	0.09
Number of days in ICU	3.0 [3.0 to 11.0]	6.0 [3.0 to 10.0]	**0.04**
ICU free days in the first 28 days	24.5 [17.0 to 25.0]	20.0 [3.0 to 24.0]	**0.003**
Mortality at day 14	2 (5.3%)	24 (16.6%)	0.08
Mortality at day 28	2 (5.3%)	30 (20.7%)	0.03

**Table 4:** Baseline biomarkers measurements.

Biomarkers	Units	0-1 co-morbidity (*n* = 38)		2 or more co-morbidities (*n* = 145)		*P* values
D-dimer	mg/L	3.2 [1.1 to 6.9]	*n* = 37	4.2 [1.8 to 9.7]	*n* = 142	0.26
Protein C	%	71.9 [46.7 to 103.4]	*n* = 37	70.8 [49.0 to 101.9]	*n* = 143	0.93
Antithrombin	%	69.0 [50.7 to 83.5]	*n* = 37	64.0 [48.8 to 80.5]	*n* = 143	0.39
Procalcitionin	ng/mL	1.0 [0.3 to 6.3]	*n* = 36	1.1 [0.4 to 5.6]	*n* = 143	0.93
CRP	mg/L	95.5 [53.0 to 199.0]	*n* = 36	106.5 [61.0 to 185.5]	*n* = 144	0.83
Fibrinogen	mg/dL	428.0 [279.7 to 596.2]	*n* = 37	394.1 [290.0 to 555.3]	*n* = 145	0.77
IL-6	pg/mL	55.4 [39.5 to 124.2]	*n* = 36	66.4 [28.3 to 226.6]	*n* = 143	0.58
Triglycerides	mmol/L	1.0 [0.6 to 1.6]	*n* = 36	1.3 [0.9 to 1.8]	*n* = 142	0.11
Cholesterol	mmol/L	2.5 [1.8 to 3.5]	*n* = 36	2.3 [1.8 to 3.4]	*n* = 143	0.54
HDL-Cholesterol	mmol/L	0.7 [0.4 to 0.9]	*n* = 36	0.7 [0.5 to 0.9]	*n* = 143	0.99
LDL-Cholesterol	mmol/L	1.5 [0.8 to 2.3]	*n* = 36	1.1 [0.6 to 2.0]	*n* = 142	0.19

## Appendix

Co-Morbidity Disease Taxonomy

Cardiac
(1) Angina
(2) Arrthythmia
(3) Valvular disease
(4) Myocardial infarction
(5) Congestive heart failure
(6) Other myocardial illness.
Vascular
(1) Hypertension
(2) 8.Peripheral vascular disease
(3) Cerebrovascular
(4) Other vascular illness.
Pulmonary
(1) Chronic obstructive pulmonary disease
(2) Asthma
(3) Other pulmonary disease.
Neurologic
(1) Dementia
(2) Hemiplegia
(3) Other neurologic illness.
Endocrine
(1) Diabetes
(2) Diabetes with end organ
(3) Other endrocrine illness.
Renal
(1) Renal disease.
Gastro-intestinal
(1) Chronic liver disease and cirrhosis
(2) Gastrointestinal bleeding
(3) Inflammatory bowel disease
(4) Peptic ulcer disease.
Cancer/immune
(1) Tumor
(2) Lymphoma
(3) Leukemia
(4) AIDS
(5) Metastatic cancer.
Miscellaneous
(1) Rheumatologic
(2) Coagulopathy
(3) Other.
